RETRACTED

# Assessment of Physical Fitness and Health Status of Athletes Based on Intelligent Medical Treatment under Machine Learning

**DOI:** 10.1155/2022/9687496

**Published:** 2022-07-30

**Authors:** Yunlong Tong

**Affiliations:** Sports institute, Jilin Normal University, Siping, Jilin 136000, China

## Abstract

Machine learning is an interdisciplinary study of how to make computer programs perform similar to human learning, and its techniques are widely used in the medical industry. The purpose of this paper is to study how to use machine learning-based intelligent medicine to analyze and study the assessment of athletes' physique and health status and describe the machine learning algorithm. This paper puts forward the problem of intelligent medical diagnosis, which is based on machine learning, and then elaborates on the concept of machine learning and related algorithms, and designs and analyzes a case of an athlete's physique monitoring and health status assessment system. The experimental results show that the athlete's physical fitness monitoring and health status evaluation system can meet the needs of users. The text classification effect based on the LSTM method is slightly inferior to the SVM effect, in which the recall rate of diabetes is not more than 40%, and the recall rate of cerebral infarction is improved by 26.5% after using fuzzy matching.

## 1. Introduction

In the 21st century, the continuous development of science and technology and intelligent computer technology has promoted the penetration of machine learning into all fields of society. China is quickly entering the era of big data, and the limits of traditional statistical analysis approaches in a variety of sectors, including medicine, are gradually becoming apparent. Intelligent diagnosis in medical treatment is also an artificial intelligence technology, a system that simulates the diagnosis experience of experts and combines the thinking process of medical knowledge. It has important uses in the medical field and has application prospects in real life.

Machine learning technology is utilized widely as we observe, in the medical industry with its powerful processing performance and decision-making capabilities. The essence of the system is to utilise the classification algorithm to develop an intelligent decision-making model based on the computer's objectivity, which can properly and effectively determine if a person has a sickness and what sort of condition they have without the need for external intervention. As a result, to lower the rate of misdiagnosis, mistakes in this decision-making process should be eliminated. Artificial intelligence technology reduces the diagnostic error rate of doctors in medical diagnosis, reduces misjudgment caused by human emotions, and can make more accurate and informed decisions than doctors. Society has entered an era of informatization and digitalization as a result of the continued growth of computer networks, and Internet+ is now widely employed in national life. The athlete's physique monitoring health assessment system organically combines the athlete's physique monitoring with Internet technology. To a certain extent, the manual processing of physical fitness monitoring data and the cumbersome statistical steps have changed, which is conducive to promoting the popularization of national monitoring.

RETRACTED

The innovation of this paper includes the following points: (1) This paper combines medical diagnosis with machine learning algorithms and introduces the theory and related methods of machine learning in detail. This paper mainly introduces principal component analysis, LSTM related technology, and support vector machine AdaBoost adaptive enhancement algorithm. (2) When faced with medical record text data, vector support machine (SVM) and LSTM are used for disease classification, respectively. By evaluating the experimental results, comparing the performance of the two methods, it is concluded that SVM is better than LSTM. After comparing the results, we found that the intelligent deep learning diagnostic capabilities of the LSTM model cannot be fully utilized when performing text analysis on electronic medical records with a small amount of data.

## 2. Related Work

In the era of big data, machine learning is a key field in the emergence of high-performance computer systems. It combines artificial intelligence and big data application technology, and it has been improved in a variety of industries. Buczak and Guven presents a concentrated literature overview of machine learning and data mining approaches that assist network analysis for intrusion detection, as well as a brief lesson for each ML/DM method. He talks on the difficulty of ML/DM algorithms and the obstacles of employing them in cybersecurity, as well as when to utilise which technique. However, the study's dataset is incomplete [1]. Mullainathan and Spiess provided a way of thinking about machine learning that has earned it a spot in the econometrics toolkit. By offering a greater understanding of how machine learning algorithms function, where they shine, and where they might go wrong, he intends to make them theoretically easier to use. He, on the other hand, overlooks the complexities of machine learning [2]. Voyant et al. described how machine learning algorithms may be used to anticipate solar radiation as well as the output power of a Solar System, which is required for a well-functioning grid or optimal energy flow management into a Solar System. Due to the variety of datasets, time steps, prediction horizons, parameters, and performance indicators, rating such approaches is difficult. His technique, on the other hand, has a low prediction performance [3]. To lead the debate of big data's benefits and difficulties, Zhou et al. presented the machine learning framework. The framework follows the preprocessing, learning, and assessment phases and is ML-centric. The stages of ML and the MLBiD components guide you in identifying relevant opportunities and problems. The paper, however, lacks a strong objective foundation [4]. Lamperti et al. specifically addressed the challenge of parameter space exploration and calibration of ABMs by combining machine learning and intelligent iterative sampling. The findings reveal that machine learning surrogates derived from the proposed iterative learning procedure are relatively accurate surrogates for genuine models. His experimental results, on the other hand, are relatively sparse [5]. Brynjolfsson and Mitchell explain what he considers to be the most important consequences for employees, as well as his criteria for what the current generation of machine learning algorithms can and cannot perform. While certain aspects of many employment are “suited for ML” (SML), other functions within these jobs are not. As a result, the impact on employment is more complicated than the straightforward substitution and substitute tale that has been highlighted by some. He did not, however, provide any explicit advice [6]. Malta et al. proposed a novel stemness measure based on the transcriptome and epigenetics of nontransformed pluripotent stem cells and their differentiated offspring to quantify the degree of nongenetic dedifferentiation. Finally, these measurements enable the discovery of new targets and potential targeted therapeutics for tumor differentiation. He did not, however, think about the method's viability [7]. Schrider and Kern talk about supervised machine learning, which is a novel paradigm in computational population genetics (ML). Finally, supervised machine learning, he believes, is an essential and neglected technique in evolutionary genomics with a lot of potential. He is not, however, grounded in reality [8].

RETRACTED

## 3. Classification Methods Based on Machine Learning

### 3.1. Definition of Machine Learning

Machine learning refers to the use of computer programs to improve the ability to judge various situations by using practical experience to improve them [9].

Typical machine learning training is mainly divided into the following processes:

1. Acquisition of datasets: the acquisition of the data set is very important. It is very important if an authoritative person instructs the collected data set to get twice the result with half the effort. Otherwise, we can only blindly analyze and detect each data characteristic, and even find the characteristic sample data set.
2. Data regularization processing: the information in the collected datasets is often very complex, including a large number of spam samples and redundant features. Therefore, it is necessary to process the data in advance to improve the availability of the data.
3. Define the training data set. The sample data such as disease diagnosis indicators are classified and standardized into a disease data set, and the disease diagnosis data set is divided into a training set and a test set according to the conventional practice in the field of disease diagnosis. The training set is used to improve the disease diagnostic model's classification accuracy, while the test set is used to assess the model's accuracy once it has been trained using real medical data.
4. The choice of classification algorithm: conventional classification methods include relatively simple fuzzy K-nearest neighbors, artificial neural networks that simulate human neurons, and random forests based on decision trees [10]. In disease diagnosis, the actual diagnosis data can be used to train different classifiers, and then the test set can be used to compare the prediction accuracy of different disease classifiers, so as to select an appropriate method, and different classifiers can also be used comprehensively.
5. Classifier training: through the samples trained by the classification algorithm, we can get a mapping of xy, which is the classification rules and mathematical rules.
6. The performance evaluation of the classifier: the ability of the classifier is judged by parameters such as error, accuracy, and scaling performance.

### 3.2. Principal Component Analysis

Principal component analysis, usually known as PCA, is a statistical methodology that uses dimensionality reduction methods to reduce data [11]. The primary goal of principle component analysis is to explain a large number of variables with a small number of variables. According to the principle of principal component analysis, the following functions can be obtained:

(1) The spatial dimension of the data can be reduced. That is, the dimension of the original data space is *X*, but the data space with dimension *Y* (*X* < *Y*) obtained after principal component analysis can replace the original data space, and the replaced data information has no or very little loss.
(2) The relationship between variables can be known.
(3) Multidimensional data can be represented by a graph. Currently, for multidimensional data with dimensions higher than 3, geometry cannot be drawn. Dimension reduction is performed by principal component analysis, and two main elements are taken, and multiple graphs can be drawn on a two-dimensional plane according to the scores of the principal components. It also provides a good method for text classification.
(4) It can be a regression model. That is, the variables after principal component analysis are used as new variables to replace the original independent variables, and regression analysis can be performed.
(5) The variables after regression analysis can be screened. Therefore, when filtering variables, the amount of calculation can be reduced to obtain the best subset of variables.
  (1) Data standardization
    (1) $$\begin{array}{c} Z_{ab}=\frac{x_{ab}-{\bar{x}}_{b}}{Q_{b}},\;a=1,2,\ldots ,n;\;b=1,2,\ldots ,m, \end{array}$$
  where, ${\bar{x}}_{b}=\left(\sum_{a=1}^{n}x_{ab}/n\right)$, $Q_{b}^{2}=\left({\sum_{a=1}^{n}\left(x_{ab}-{\bar{x}}_{b}\right)}^{2}/n-1\right)$.
  (2) Calculate the correlation coefficient matrix
    (2) $$\begin{array}{c} G={\left[g_{ab}\right]}_{m}xm=\frac{Z^{V}Z}{n-1}, \end{array}$$
  among them, *g*_*ab*_=(∑*Z*_*cb*_*Z*_*cb*_/*n* − 1)*a*, *b*=1,2,…, *m*.
  (3) Solve the matrix to determine the number of principal components
    (3) $$\begin{array}{c} \left|G-\beta I_{m}\right|=0, \end{array}$$
    (4) $$\begin{array}{c} \frac{\sum_{b=1}^{d}\beta_{b}}{\sum_{b=1}^{m}\beta_{b}}\geq 0.85. \end{array}$$
  Solve (3) to get the characteristic root of the Formula, determine the value of *d* in formula (4), find the Formula *Gb*=*β*_*b*_*e* of each *β*_*b*_, *b*=1,2,…, *d*, and get the characteristic vector *e*_*b*_^*o*^.
  (4) Principal component generation
    (5) $$\begin{array}{c} R_{ab}=Z_{a}^{V}e_{b}^{o},\;b=1,2,\ldots ,d. \end{array}$$
  Among them, *R*_1_, *R*_2_, and *R*_3_ are the first, second, and third principal components, and so on, *R*_*d*_ is the d-th principal component.
  (5) Principal component evaluation

For d-th *R*_1_, *R*_2_,…, *R*_*d*_, the principal components are first weighted and then summed to obtain the evaluation value, in which the variance contribution rate is the weight.

RETRACTED

### 3.3. LSTM-Related Technologies

LSTM neural network is a variant of recurrent neural network. It mainly adds a Forget Gate on the basis of RNN to solve the long-distance dependency problem of RNN. The purpose of the hidden layer block is to use these three “gates” to limit whether the data information can be filtered (i.e., added or deleted) through the Cell. At present, the names of these three effective “gates” are: input gate, forget gate, and output gate [12, 13]. The functions of these three “doors” are described in detail.

#### 3.3.1. Forgotten Gate

The main function of the forget gate is to decide whether to keep or delete the previous data information. It first sets two parameters: “0” and “1” (“0” means to leave data information, “1” means to delete data information), and then calculate the input of the two-time states to obtain a value between the two parameters. Finally, it is used on the Cell at the last moment to judge whether the data information of the last two moments is left or deleted.

#### 3.3.2. Input Gate

The main function of the input gate is to judge whether the input data information is allowed to be updated to the Cell, so as to filter and adjust some unnecessary information. It first sets two parameters: “0” and “1” (“0” means that data information cannot pass through, and “1” means that data information can pass through). Then use the sigmoid function to calculate the value, and this value is between the two parameters, and finally use the data information at the time of input to determine whether the input data is passed, and whether it is updated to the Cell state.

#### 3.3.3. Output Gate

The main function of the output gate is to determine whether the conditions are met to output based on the value of the Cell state and the value obtained after data processing. It first sets two parameters: “0” and “1” (“0” means that the data information is not allowed to be output, and “1” means that the data information is allowed to be output). Then calculate the value obtained based on the current state of the Cell to determine whether the output is allowed to be output.

The LSTM model structure is shown in Figure 1.

From Figure 1, we can see that the network structure constructed in this paper contains three layers: input gate, forget gate, and output gate. And through the control of the three gates, it has an effect on the Cell structure. It is not difficult to see that the output gate, forget gate, and input gate of the three layers of the mechanism have the same input [14].

That is, the same has the following three items:

  Input 1: we denote the output at the previous time node as *e*_*h*′_, which is used to represent the output of the node at position *h*′ at the previous time node
  Input 2: the input of the current LSTM block unit is denoted as *Q*_*c*′_, which represents the input of the i-node at the block position of the block unit
  Input 3: denote the Cell state of the LSTM subunit at the previous time as *Q*_*c*′_, which is used to represent the Cell value of the *c*′ node at the previous time position

However, there are four inputs to the Cell state of the LSTM subunit:

  Input 1: the input 1 of the Cell state of the LSTM subunit is the same as the input 1 of the output gate, forget gate, and input gate.
  Input 2: the input 2 of the Cell state of the LSTM subunit is the same as the input 2 of the output gate, forget gate, and input gate.
  Input three: different from the output gate, forget gate, and input gate mentioned, the same input three. It is to denote the output of the forget gate at the same moment in the unit block as *n*_*f*_, which is used to represent the value of the f-th node of the forget gate at the current moment.
  Input 4: it is one more input than the output gate, forget gate, and input gate. It is to denote the output of the input gate at the same time in the unit block as *n*_*j*_, which is used to represent the value of the jth node of the input gate at the current time.

RETRACTED

Therefore, according to the role and relationship between the mentioned three “gates” and Cell, Figure 2 is obtained based on the connection between input and output.

According to the Figure, the calculation formulas of the three “gates” and the LSTM subunit Cell at the time *t* node can be found.

Enter the gate calculation formula:

(6) $$\begin{array}{c} m_{j}^{t}=\sum_{i=1}^{I}W_{ij}O_{i}^{t}+\sum_{h^{\prime }}^{H}W_{h^{\prime }j}n_{h^{\prime }}^{t-1}+\sum_{a^{\prime }=1}^{A}W_{a^{\prime }j}Q_{a^{\prime }}^{t-1}, \end{array}$$

(7) $$\begin{array}{c} n_{j}^{t}=f\left(m_{j}^{t}\right). \end{array}$$

The forget gate calculation formula:

(8) $$\begin{array}{c} m_{f}^{t}=\sum_{i=1}^{I}W_{if}O_{i}^{t}+\sum_{h^{\prime }}^{H}W_{h^{\prime }f}n_{h^{\prime }}^{t-1}+\sum_{a^{\prime }=1}^{A}W_{a^{\prime }f}Q_{a^{\prime }}^{t-1}, \end{array}$$

(9) $$\begin{array}{c} n_{f}^{t}=f\left(m_{f}^{t}\right). \end{array}$$

Through the two formulas, it is found that the input gate and the forgetting gate are actually the same.

Cell state calculation formula:

(10) $$\begin{array}{c} m_{a}^{t}=\sum_{i=1}^{I}W_{ia}O_{i}^{t}+\sum^{H}W_{h^{\prime }a}n_{h^{\prime }}^{t-1}, \end{array}$$

(11) $$\begin{array}{c} n_{a}^{t}=G\left(m_{a}^{t}\right), \end{array}$$

(12) $$\begin{array}{c} Q_{A}^{t}=n_{f}^{t}Q_{a^{\prime }}^{t}+n_{j}^{t}n_{a}^{t}. \end{array}$$

Output gate calculation formula:

(13) $$\begin{array}{c} m_{w}^{t}=\sum_{i=1}^{I}W_{iw}O_{i}^{t}+\sum_{h^{\prime }=1}^{H}W_{h^{\prime }w}n_{h^{\prime }}^{t-1}+\sum_{c=1}^{A}W_{aw}Q_{a^{\prime }}^{t-1}, \end{array}$$

(14) $$\begin{array}{c} n_{w}^{t}=f\left(m_{w}^{t}\right). \end{array}$$

The difference between the output gate and the input gate and the forget gate is the Cell state value to the current time point.

RETRACTED

The final output is

(15) $$\begin{array}{c} n_{h}^{t}=n_{w}^{t}H\left(Q_{a}^{t}\right). \end{array}$$

### 3.4. Support Vector Machines

The Support Vector Machine (SVM) is designed to be extended to the nonlinear field according to the linear classification by using statistical theory. The multi-bit surface constructed by the model maximizes the Euclidean distance between the samples of different categories and the solution surface. As researchers continue to expand the application field of SVM, SVM can also be used to solve traditional problems such as excessive problem solution space and overlearning. In both academia and industry, SVM has made great progress in the theoretical research and practical application. SVM, its theoretical basis is the VC dimension theory of statistical learning, is that the error rate on the limited sample test set is bounded by the sum of the terms associated with the VC dimension of the training error rate [15]. When faced with these limited data samples that can be separated, the value of the training error rate is zero at this time, and the value of structural risk is guaranteed to be minimized.

The AdaBoost adaptive boosting algorithm learns by combining multiple classifiers (such as SVM and KNN) using actual training data. Its adaptive performance is to weight the previous misclassified samples and then use these weighted samples to train the next base classifier and at the same time add new classifiers [16].

That is to say, the entire AdaBoost iterative algorithm is divided into three steps:

1. Assign weights to the sample data in each training set, and the setting of the weights is determined according to the field and experience, for example, it is directly set as the reciprocal of the number of sample data.
2. Train a weak classifier. If in the process, some samples have been classified more accurately, and then in the next training set, the weight will be reduced. All samples with reduced weights are used in the next classifier, and so on.
3. Combine the obtained classifiers into a strong classifier. Then, after the training of multiple weak classifiers is completed, the weight of each classifier in the combined total classifier is determined according to the classification error of each classifier. The ultimate purpose is to supervise the overall classifier error and improve the accuracy.

*T*={(*a*_1_, *b*_1_), (*a*_2_, *b*_2_) … (*a*_*N*_, *b*_*N*_)} is a set of training data, instance *a* ∈ *A*, instance space *A* ∈ *Q*^*n*^, and *b*_*i*_ belong to the set {−1,+1}. AdaBoost learns weak or basic classifiers from training data and combines them into a powerful classifier as follows:

First, initialize the weight distribution of the training data, giving each sample the same weight: 1/N.

(16) $$\begin{array}{c} Z_{i}=\left(s_{11},s_{12}\ldots s_{1i},s_{1N}\right),\;s_{1i}=\frac{1}{N},\;i=1,2,\ldots . \end{array}$$

Then iterate, use *c*=1,2, .., C to display the number of iterations to the round.

(a) Use the weighted *Z*_*c*_ training dataset to learn to obtain the basic classifier
  (17) $$\begin{array}{c} O_{c}\left(a\right):\chi ⟶\left\{-1+\right.. \end{array}$$
(b) Calculate the *O*_*c*_(*a*) error rate
  (18) $$\begin{array}{c} e_{c}=P\left(O_{c}\left(a_{i}\right)\neq b_{i}\right)\\ =\sum_{i=1}^{N}s_{ci}I\left(O_{c}\left(a_{i}\right)\neq b_{i}\right). \end{array}$$
The setting of these formulas is based on the error rate *e*_*c*_ of the i-th model *O*_*c*_(*a*_*i*_) in the training set to determine the weights.
(c) Calculate the coefficient of each model *O*_*c*_(*A*_*i*_), *α*_*c*_ indicates the importance of *O*_*c*_(*A*)
  (19) $$\begin{array}{c} \alpha_{c}=\frac{1}{2}\log\frac{1-e_{c}}{e_{c}}. \end{array}$$
Among them, when the error rate is lower than 0.5, the importance of the model decreases monotonically with the error rate, thus achieving the purpose of combining the models and the importance of the model with a small error rate becomes greater.
(d) Update the weights for the next round of iteration
  (20) $$\begin{array}{c} Z_{c+1}=\left(s_{c+1,1},s_{c+1,2}\ldots s_{c+1,i}\ldots ,s_{c+1}s_{c+1,i}\right)\\ =\frac{s_{ci}}{D_{c}}\exp\left(-\alpha_{c}b_{i}O_{c}\left(a_{i}\right)\right),\;i=1,2,\ldots ,N. \end{array}$$

Increase the weight of misclassified samples and decrease the weight of correctly classified samples on the base classifier *O*_*c*_(*A*). Using this method, AdaBoost can focus on hard samples.

RETRACTED

*D*_*c*_ is the normalization factor, making *D*_*c*+1_ a probability distribution

(21) $$\begin{array}{c} D_{c}=\sum_{i=1}^{N}s_{ci}\exp\left(-\alpha_{c}b_{i}O_{c}\left(a_{i}\right)\right). \end{array}$$

Finally, combine the individual weak classifiers

(22) $$\begin{array}{c} f\left(a\right)=\sum_{c=1}^{C}\alpha_{c}O_{c}\left(a\right). \end{array}$$

Thus, the final classifier is obtained as follows:

(23) $$\begin{array}{c} O\left(a\right)=\text{sign}\left(f\left(a\right)\right)\\ =\text{sign}\left(\sum_{c=1}^{C}\alpha_{c}O_{c}\left(a\right)\right). \end{array}$$

Adaptive augmentation algorithms are rarely used in regression problems. Different combination strategies of various adaptive enhancement methods can be used to solve two-class problems, multi-class problems, etc. In practice, each training sample in the training set will be used to train the overall model.

## 4. Experiment and Analysis of Intelligent Medical Treatment for Physical Fitness Monitoring and Health Assessment of Athletes

### 4.1. Applicability of Machine Learning Algorithms in Intelligent Medical Diagnosis

In the classification stage, we try to apply machine learning techniques (i.e., SVM algorithm) to learn classification of the labeled feature vectors. At the same time, the performance of these two machine learning algorithms in the application of intelligent medical diagnosis assistance is evaluated and analyzed, and the classification effect of the popular deep learning classification method and the machine learning classification method is used to compare the classification effect [17].

RETRACTED

In the same text, perform feature extraction, rank high-frequency words, and then conduct experiments.

#### 4.1.1. Experimental Results Based on SVM Classification Algorithm

We used the 1-v-1 SVMs method to design an SVM between any two classes, and a total of three SVMs were designed for 1400 cases of diabetes, 700 cases of cerebral infarction, and 1300 cases of chronic obstructive pulmonary disease.

The test also has different results according to the matching mode during word segmentation, and the evaluation criteria are precision and recall.

Accuracy (Precision) = number of correct classification/number of positive cases.

Recall rate (Recall) = number of correct classification/total number of positive examples.

The F1 value is the harmonic mean of the two.

When designing the SVM applied to diabetes classification, we used 1400 cases of diabetes as training positive samples, the remaining 1800 cases of diseases as training negative samples, and the remaining 500 cases of diabetes and 600 cases of other diseases as test sets. When designing the SVM applied to the classification of cerebral infarction, it is considered that there are only 700 cerebral infarction cases and 2600 negative examples. In order to avoid the imbalance of the data set, we randomly selected 1000 cases out of 2600 cases, of which 700 cases were used as training set and 300 cases were used as test set. Among the 700 cases of cerebral infarction, 550 cases were randomly selected as training set and 150 cases were used as test set. In designing SVMs applied to the classification of chronic obstructive pulmonary disease. We randomly select 1,000 of the 1,300 cases as the training set, the remaining 300 as the test set, and among the negative examples, 2,000 as the training set and 300 as the test set.

The results obtained from experiments are shown in Figure 3.

The experimental results show that fuzzy matching can effectively improve the accuracy when there are more positive examples than negative examples, while the recall rate and F1 value will decrease. The disease with the best classification effect is cerebral infarction, while the classification effect of chronic obstructive pulmonary disease is relatively low.

RETRACTED

#### 4.1.2. Experimental Results Based on LSTM Classification Algorithm

The division of training set and test set is the same, and the experimental results we get are shown in Figure 4.

From the experimental results, the text classification effect based on LSTM method is much worse than that of SVM. Especially the recall rate, in which the recall rate of diabetes is not more than 40%, and the recall rate of cerebral infarction is improved by 26.5% after using fuzzy matching. It can be seen that the LSTM method failed to successfully learn the disease classification experience of human doctors. Small sample data cannot build deep learning models.

### 4.2. Athlete Physical Fitness Monitoring Health Evaluation System Database

In the user information table, the basic information of the user is mainly stored. Due to the privacy of physical fitness monitoring information, in order to ensure the information security of each user, users must register on this website and log in correctly to view basic user information [18, 19]. The user then selects Login after entering his or her username and password. The system then goes back to the database's user information table and checks the data in the table with the information supplied by the user. Only after a successful comparison may the user data be used. The specific data of this information table are shown in Table 1.

The user reservation table saves the information of the current reservation user. Whenever a user has successfully made an appointment for physical fitness monitoring, the system will automatically record the specific information of the user's appointment into the user appointment form, which is convenient for the system administrator to query. The user reservation form includes the basic information of the user, the reservation time for physical fitness monitoring, the reserved physical fitness monitoring organization, and the reserved items. In the appointment item, 0 means no appointment, 1 means appointment, if the appointment item field is empty, no appointment is made by default. The specific information in the user reservation table is shown in Table 2.

The information of each physical examination of the user is saved in the user's physical fitness monitoring table. After the user's physical examination is completed, the physical fitness monitoring results can be uploaded, and the athlete physical fitness monitoring health assessment system will give corresponding scores and evaluation levels according to the user's physical fitness monitoring results. The user physique monitoring table is shown in Table 3.

RETRACTED

In the physical fitness monitoring scoring table, the scoring standards of the “National Physical Fitness Measurement Standards” are stored. This table is a scoring table for the user's physical fitness monitoring. After the user completes the physical fitness monitoring, the system will compare the results of the physical fitness monitoring with the physical fitness monitoring scoring table, and finally obtain the corresponding score [20]. The system administrator can modify and update the table according to the “National Physical Fitness Determination Standard” promulgated by the State Sports General Administration. The specific content of the physical fitness monitoring score table is shown in Table 4.

In the athlete physique health assessment system, in order to ensure the privacy of user information, certain settings are made for external access to the athlete physique health system. The specific process is shown in Figure 5.

In the user registration and login stages of the athlete physique monitoring and health assessment system, it is first necessary to verify and filter the information entered by the user. Because there are some users in the network at present, they try to invade the system database by entering special command statements in the external interface of the system database, so as to realize the purpose of illegally browsing the database data [21–23]. The user name and password that the user must input when checking in to the athlete physique monitoring health assessment system are the two most common external database interfaces. During the login and registration processes, users of the athlete physique monitoring and health assessment system must interact with the system database. Therefore, in order to prevent illegal intrusion, it is first necessary to filter and check the data input by the user of the athlete physique monitoring and health assessment system. Secondly, the athlete fitness monitoring health assessment system will perform a one-way encryption operation on the password entered by the user [24, 25]. One-way encryption is a cryptographic technique that cannot be reversed. Some unauthorised users log in using other people's usernames and passwords in order to prevent data leakage in the database of the athlete's physical fitness monitoring and health assessment system, causing personal information and health data to be released. A one-way encryption mechanism is used to encrypt and preserve the user password in the athlete physique monitoring and health evaluation system. Even if the athlete's physical fitness monitoring and health assessment system's database is unlawfully accessed, the illegal user will not be able to gain the user's account password, which safeguards the user's information to some extent. When a user logs in, the password entered by the user must likewise be encrypted, and the encrypted cipher text of the password must then be directly compared to the true password.

RETRACTED

### 4.3. Realization and Optimization of the Physical Fitness Assessment System for Athletes

For an athlete fitness monitoring health assessment system, a connected mode is required. The login feature allows websites to accurately authenticate users [26, 27]. When users visit the site, they can register and log in, while also disconnecting the user's logged-in state keeping user data safe [28–30]. The specific process and login diagram are shown in Figures 6 and 7.

After correctly logging in to the National Physical Fitness Monitoring Health Assessment System, users can view all relevant information in the system, including appointmentable monitoring agencies, appointmentable items and time. Each monitoring agency in the athlete fitness monitoring and health assessment system has an upper limit for the number of appointments. If the upper limit is reached within a certain period of time, the agency will no longer be able to accept appointments. In the physical fitness monitoring appointment, the user can select the time, item, and institution of physical fitness monitoring. The system will automatically determine whether the reservation is successful according to the actual situation of the institution. If successful, the reservation information will be stored in the database. If it fails, the reason for the failure will be returned so that the user can modify it accordingly. The specific operation process is shown in Figure 8.

After the user performs physical fitness monitoring at the institution, he or she can choose to have the institution input the monitoring data on its behalf or by itself. Input the data into the athlete's physical fitness monitoring health evaluation system so that the athlete's physical fitness monitoring health evaluation system can make a correct evaluation of the user's physical fitness monitoring results. When the physical fitness monitoring results are input, the input data will also be checked to ensure the validity of the input data and prevent mis-input. After the physical fitness monitoring results are entered into the website, users can log in to the website anytime and anywhere to view the monitoring data. The specific process is shown in Figure 9.

The athlete's physique monitoring and health assessment system has formulated a systematic scoring standard according to the “National Physical Fitness Measurement Standard” promulgated by the State Sports General Administration. After the physical fitness monitoring is completed, the user submits the monitoring results to the athlete physical fitness monitoring health assessment system, and the system will compare the monitoring results with the “National Physical Fitness Measurement Standards” to obtain corresponding scores. A total of 300 athletes were selected for physical fitness monitoring and evaluation in this experiment. Among them, there are 100 female athletes and 200 male athletes. The results are shown in Figures 10 and 11.

RETRACTED

According to the test case of the national physique monitoring health assessment system, the system has been tested. The test results show that, according to the test cases of the national physique monitoring and health assessment system, most of the functional modules test whether each functional module of the system can run normally. Among them, athletes with a height of 5 points accounted for the most, with a total of 98.67%.

## 5. Discussion

First of all, through the study of relevant knowledge points of literature works, this paper initially masters the relevant basic knowledge and analyzes how to study the assessment of athletes' physique and health status based on intelligent medical treatment based on machine learning. In addition, the paper expounds the concepts of machine learning and related technical algorithms, focuses on the research on LSTM related technologies, and explores the application of AdaBoost adaptive enhancement algorithm in support vector machines. And it analyzes the applicability of machine learning algorithms in intelligent medical diagnosis through experiments and constructs an athlete's physical fitness monitoring and health assessment system.

This paper also focuses on the introduction of the LSTM neural network as a variant of the recurrent neural network. The block unit of the hidden layer is the most important, which is constructed with three “gate” designs. Support vector machines have made great progress in the theoretical research and practical application of SVM in academia and industry. With the entry into a new era, the continuous development of intelligent computer technology has promoted the wide application of machine learning in various fields of life.

Through the experimental analysis in this paper, we can see that the text classification effect based on the SVM method is better than that of the LSTM method. The LSTM method fails to successfully learn the disease classification experience of human doctors, and the deep learning model cannot be constructed with small sample data. In the athlete physique monitoring health assessment system, system users can subscribe to physique monitoring and search results through the system. They can easily understand their fitness level by displaying relevant fitness monitoring reports and comparing their own results. At the same time, it also provides a publicity channel for the country to promote national fitness.

RETRACTED

## 6. Conclusion

With the rapid development of the current era and the rapid progress of science and technology, the importance of machine learning in medical diagnosis is becoming more and more obvious. Artificial intelligence and natural language processing technology have been advancing, and intelligent diagnosis will be more deeply embedded in the lives of the public. The athlete's physical fitness monitoring and health assessment system has played a certain role in promoting national fitness and the popularization of physical fitness monitoring and has changed the tedious steps of artificial physical fitness monitoring and statistics in the past. Through the Internet and database technologies, it realizes the automation of data statistics, the popularization of athlete monitoring, and the simplification of result query. In this paper, machine learning and medical diagnosis are organically integrated, and the designed athlete physique monitoring health assessment system has realized most of the required functions in the athlete physique monitoring. However, there are still many parts that need to be improved in this paper, such as how the system can provide users with functions such as health improvement plans, which need to be improved in future work.

## Figures and Tables

**Figure 1:** LSTM hidden layer block.

**Figure 2:** The relationship between the three “gates” and Cell.

**Figure 3:** Experimental results with and without fuzzy matching for three diseases (a) Use fuzzy matching; (b) do not use fuzzy matching.

**Figure 4:** Experimental results with and without fuzzy matching for various diseases (a) Use fuzzy matching; (b) do not use fuzzy matching.

**Figure 5:** System security control flow.

**Figure 6:** System user login flowchart.

**Figure 7:** System user login page.

**Figure 8:** System user reservation process.

**Figure 9:** Process of physical fitness monitoring results.

**Figure 10:** Physical fitness monitoring and assessment of female athletes.

**Figure 11:** Physical fitness monitoring and evaluation of male athletes.

**Table 1:** User information form.

The serial number	The field name	Field meaning	Length	The data type	Whether empty
1	user_id	User ID, primary key	11	int	No
2	user_login	The user name	20	varchar	No
3	user_password	Password	8	varchar	No
4	user_name	The name	20	varchar	No
5	user_sex	Gender	20	varchar	Yes
6	user_birthday	Date of birth		date	Yes
7	user_age	Age	8	int	No
8	user_group	Nation	20	varchar	Yes
9	user_occupation	Occupation	255	varchar	Yes
10	user_contact	Contact information	255	varchar	Yes

RETRACTED

**Table 2:** User appointment form.

The serial number	The field name	Field meaning	Length	The data type	Whether empty
1	appointment_id	Reservation number	11	int	No
2	appointment_user	Reservation user ID	11	lnt	No
3	appointment_company	Monitoring organization ID	11	int	No
4	appointment_date	Time of appointment		date	No
5	appointment_height	Height	4	int	Yes
6	appointment_weight	Weight	4	int	Yes
7	appointment_vc	Vital capacity	4	int	Yes
8	appointment_step	Step test	4	int	Yes
9	appointment_sitandReach	Sitting and standing early flexion	4	int	Yes
10	appointment_jump	Standing long jump			Yes
11	appointment_grip	Grip strength test	4	int	Yes
12	appointment_situp	Abdominal curl	4	int	Yes

**Table 3:** User physical fitness monitoring table.

The serial number	The field name	Field meaning	Length	The data type	Whether empty
1	test_id	Monitoring number	11	int	No
2	test_user	Monitor user ID	11	lnt	No
3	test_company	Monitoring organization ID	11	int	No
4	test_date	Monitoring time		date	No
5	test_height	Height	100	varchar	Yes
6	test_weight	Weight	100	varchar	Yes
7	test_vc	Vital capacity	100	varchar	Yes
8	test_step	Step test	100	varchar	Yes
9	test_sitandReach	Sitting and standing early flexion	100	varchar	Yes
10	test_jump	Standing long jump	100	varchar	Yes
11	test_grip	Grip strength test	100	varchar	Yes
12	test_situp	Abdominal curl	100	varchar	Yes

**Table 4:** Physical fitness monitoring score table.

The serial number	The field name	Field meaning	Length	The data type	Whether empty
1	score_id	Monitoring number	11	int	No
2	score_item	Monitoring name	100	varchar	No
3	score_level1	Level 1	100	varchar	Yes
4	score_level1up	Level 1 upper bound	100	varchar	Yes
5	score_level1down	Level 1 lower bound, level 2 upper bound	100	varchar	Yes
6	score_level2	Level 2	100	varchar	Yes
7	score_level2down	Level 2 lower bound, level 3 upper bound	100	varchar	Yes
8	score_level3	Level 3	100	varchar	Yes
9	score_level3down	Level 3 lower bound, level 4 upper bound	100	varchar	Yes
10	score_level4	Level 4	100	varchar	Yes
11	score_level4down	Lower bound of level 4	100	varchar	Yes

## Data Availability

Data sharing is not applicable to this article as no new data were created or analyzed in this study.
